The article "Development Analysis of the Sports Industry Based on the Data Mining Model" was published in 2022. Journal: Comput Intell Neurosci.

# Development Analysis of the Sports Industry Based on the Data Mining Model

**DOI:** 10.1155/2022/7543957

**Published:** 2022-06-29

**Authors:** Qi Huang, Xiaowei Zou, Tao Zhang, Haidong Yang

**Affiliations:** ^1^Department of Physical Education, Heilongjiang Bayi Agricultural University, Daqing, Heilongjiang 163319, China; ^2^College of Humanities and Social Sciences, Heilongjiang Bayi Agricultural University, Daqing, Heilongjiang 163319, China; ^3^College of Landscape Architecture and Horticulture, Heilongjiang Bayi Agricultural University, Daqing, Heilongjiang 163319, China; ^4^Canada Software Development Co. Ltd., Québec 999040, Canada

## Abstract

The Chinese sports industry encompasses both the secondary and tertiary sectors of the country's economy. More prominent are the issues of unbalanced industrial structure development, mismatch between supply and demand, and rapid expansion of the sports goods manufacturing industry. This paper first employs the literature method to investigate the dynamic mechanism and promotion strategy of China's sports industry's green development. In order to improve the accuracy of data mining and quantitative analysis in the sports industry, this paper proposes a time series-based model for the analysis of sports industry data. Utilizing the global steady-state feature fusion method, the statistical and quantitative fusion analysis method, and the fuzzy analytical control method, accurate mining of sports industry data is achieved. The simulation results demonstrate that this method has greater precision and a higher degree of feature matching for sports industry data mining, thereby reducing the disturbance error of sports industry data mining.

## 1. Introduction

China has unveiled the green development engine, which requires the country to adhere to green development principles and promote the building of a beautiful China. Green growth in economic development is defined as the symbiotic, integral, and coordinated development of the economic system, the social system, and the natural system, where the economic system is based on green growth, i.e., production and consumption are characterized by low energy consumption, low material consumption, and low emissions, in order to achieve economic growth and energy decoupling [1, 2]. According to the Marxist concept of development, green growth investigates the origins of problems, focusing on the reevaluation, and modification of the interaction between humans and their natural environment. The control of the entire consumption process necessitates an immediate transformation of the current extensive production system and way of life. Thus, green development is a constraint on the production and consumption of all industrial systems in the national economy and a prerequisite for transition from an extensive to an intensive mode of development. As a result of the green development of the sports industry, we must view it as a fundamental precondition for advancing the sports industry of my country towards high-quality development. To continuously reduce the energy consumption, material consumption, and carbon emissions produced by various categories of the sports industry, it is necessary to optimize the industrial structure, accelerate the transformation and upgrading of production methods, improve the green construction standards of sports venues, and utilize technological innovation and compensation measures to their fullest extent [3, 4].

The article "Development Analysis of the Sports Industry Based on the Data Mining Model" was published in 2022. Journal: Comput Intell Neurosci.

The sports industry in my country is a comprehensive industry that includes both secondary and tertiary industries, and it is expanding rapidly. It is becoming more difficult to address the issues of uneven industrial structure development, mismatch between supply and demand, and expansive growth in the sports goods manufacturing industry. In addition, the current internal industrial structure of the sports service industry is unworkable, as the vast majority of the industry's output is still based on primary services and is closely tied to the production of sporting products. The output scale in the high-end sports service industry equals the sum of the input scales for information technology, capital, intelligence, and talent. Consequently, the sports service industry is under increasing pressure to optimize its structure and transform into a more capital- and knowledge-intensive sector [5–7]. In conjunction with the industrial reality of the gray development of major stadiums, we must consider the long-term development of the sports sector from the standpoint of green development and environmental sustainability. Based on current and historical data, it appears that the sports business has maintained strong growth in the past and will continue to have significant opportunity for expansion in the future. In order to meet the growing need for high-quality development in the sports sector, it is more vital than ever to adhere to green development principles throughout the industry's linear growth process.

A big data fusion and a characteristic mining model for the sports industry will be developed as a result of the integrated development of the sports industry, which will allow for further organized integration and scheduling of the sports industry in the information environment. Establishing a sports industry data accurate mining model based on the information distribution of the sports industry, combined with statistical analysis and integrated scheduling methods, improves the sports industry's big data sharing and information scheduling capabilities, in order to enhance the sports industry's structural integration and development capabilities, and conducting relevant sports industry data mining model research on the optimization, upgrading, and integrating [8–14].

The article "Development Analysis of the Sports Industry Based on the Data Mining Model" was published in 2022. Journal: Comput Intell Neurosci.

According to the findings of the research, an accurate mining model for sports industry data can be developed by analyzing the peculiarities of the sports industry's big data chain. In the context of big data and cloud platform analysis, it is necessary to analyze and control, establish a green industry chain that meets the development needs of the sports industry, and design an accurate mining model for the sports industry in order to improve the accuracy of sports industry data mining ability. The design approaches for an accurate mining model of sports industry data in the traditional method are mostly comprised of the vector regression analysis method, spatial information fusion method, statistical analysis method, and ambiguity detection method [15–19]. It is possible to obtain accurate mining of sports industry data, although the accuracy of traditional methods of sports industry data mining is not very high.

In light of the inadequacies of previous methods, this study presents a time series-based strategy for developing a precise sports data mining model. To build a distributed time series model of sports industry data, the global steady-state feature fusion method is employed first, followed by the statistical and quantitative fusion analysis method, which is used to realize the quantitative spatial transformation of sports industry data features. Using the output gain steady-state analysis method, a linear analytical parameter analysis model for sports industry data mining is then constructed. Utilizing square programming and linear fusion techniques, sports industry data mining achieves endogenous fusion and parameter control, respectively. Linear clustering processing of statistical characteristics of data from the sports industry is quite effective when combined with fuzzy clustering. It is possible to design a time fusion sequence for sports industry data mining when the sparse feature matching scheduling model is used in conjunction with it, and accurate mining of sports industry data can be achieved through time series reconstruction. At the conclusion of the study, simulation test analysis is conducted, which demonstrates that the method presented here has superior performance in terms of enhancing the ability to extract accurate information from sports sector data.

The article "Development Analysis of the Sports Industry Based on the Data Mining Model" was published in 2022. Journal: Comput Intell Neurosci.

## 2. Background and Development Proposals

### 2.1. Problems

The sporting goods manufacturing industry has the critical responsibility of fostering the expansion of the sports market, increasing the availability of sports goods, and ensuring the industry's continued existence. In addition to gaining a great deal of manufacturing expertise and experience over the past few decades, it has also produced a vast quantity of primary goods to meet specific social demands. As a result of the overall expansion of the China's secondary sector, the manufacturing of sporting goods and related items is deeply intertwined with the business model of primary product processing and production, and the development of industries with a high added value is woefully behind the times. The total output of the sports goods manufacturing industry has increased from 1,123.8 billion yuan in 2015 to 1,361.4 billion yuan in 2019, and thanks to the government's continued support for the sports industry and its rapid development. This represents an average annual growth rate of only 5.3%, which is significantly lower than the national average of 7.3%. In recent years, the sports industry and the national economy's GDP growth rate have both slowed as a result of the inflationary factor. During this period, the real growth rate of the sports goods manufacturing industry has also slowed. Likewise, the athletic goods manufacturing industry is still in its nascent stages of growth. As a result of the change in the country's factor structure, the broad development model of the athletic goods manufacturing industry can no longer meet the fundamental criteria of the country's ecological civilization construction, according to some researchers who had a negative impact [20].

Developing the consumer service industry is an efficient means of upgrading the consumption structure of urban and rural residents, enhancing people's livelihood and well-being, and better addressing the growing demands of people for better living foundation. Although the daily sports service industry includes a variety of sub-businesses, such as sports fitness and leisure services, sports competitions and performances, sports venue facilities services, sports education and training, and sports tourism services, it is responsible for radiating all of the people's sports fitness, venue security, competition viewing, and a variety of important links, such as health care and leisure. In 2019, total output of the sports service industry was 846.4 billion yuan, accounting for 12% of total output in the industry in 2019. Ontology industries, such as sports competitions and performances, in particular, require urgent improvement in terms of their degree of industrialization, which must be addressed immediately. Apart from serving the demands of the public and creating economic benefits, the sports service business is also under increasing pressure to promote environmental friendly and low-carbon development. Because of the large body mass and internal space requirements of stadiums, as well as the specific environmental requirements of sports competitions, stadiums will generate a significant amount of greenhouse gases in order to meet the parameters requirements of athletes and spectators, such as light, heat, and environmental humidity during operation.

The article "Development Analysis of the Sports Industry Based on the Data Mining Model" was published in 2022. Journal: Comput Intell Neurosci.

### 2.2. Development Mechanism

With regard to industrial development, the term “dynamic mechanism” is most commonly used to refer to a dynamic system formed by the interaction and mutual influence of various internal and external forces during the course of industrial development in order to continuously promote the achievement of goals. A number of elements contribute to the driving force for the green growth of the sports industry, and various factors combine to form the driving force for the green development of the sports industry as a result of their interconnection and interaction. In accordance with general laws of industrial development and current situation in the sports industry, this research establishes the bottom-line binding force of the concept of green development, the driving force for high-quality development in the sports industry, the driving force for the integrated development of digital technology and the sports industry, and the driving force for the increase in the competitiveness of sports businesses. Green development is the primary content of the dynamic mechanism of the sports industry's green development dynamic mechanism [21].

While binding force originated as a legal notion, it has since become frequently employed in social scientific research to emphasize the restrictions or regulation of pertinent applicable issues such as methods, systems, procedures, and concepts that are important to the study at hand. The notion of green development demonstrates the dialectical and unified relationship that exists between ecological environmental protection and economic and social growth in a profound and meaningful way. It is the culmination of China's experience in dealing with the relationship between economic development and ecological environmental protection, and it is the most fundamental requirement for industrial economic development and ecological balance in the new development stage of the country's development. A critical component and fundamental requirement of high-quality development, green development is the whole limitation on all industrial elements of the national economy, and the sports industry, which has experienced rapid growth in recent years, does not constitute an exception to this. Compared to 2006, the entire size of the China's sports sector has increased from 301.1 billion yuan to 2,948.3 billion yuan in 2019 (see chart below). During this time period, the industry has witnessed significant expansion and is expected to reach a scale of approximately 5 trillion yuan by 2025. Some academics anticipate that the added value of the China's sports sector would approach 8 trillion yuan by 2035 and that the proportion of the added value of the sports industry to GDP will exceed by 4 percent. Consequently, because the sports industry possesses the characteristics of a complex industry, it is essential that it adhere to the general requirements of the coordinated development of economic growth and the ecological environment, i.e., in order to achieve linear growth in the sports industry, it is essential that it adhere to the bottom-line constraints of environmental friendly development.

The article "Development Analysis of the Sports Industry Based on the Data Mining Model" was published in 2022. Journal: Comput Intell Neurosci.

Integration of digital technology and the sports industry has emerged as the primary and most potent driving force for the development of the sports industry in general and the sports industry in particular. The use of digital technology to promote the green and low-carbon growth of the sports business has the potential to be highly effective. Based on digital technology, the digital economy offers several advantages over traditional economic activity, including faster market response, lower marginal costs, less resource consumption, and less environmental impact. The digital economy offers numerous benefits, such as innovation, environmental friendliness, and sharing, which are all compatible with the new development model. It has the potential to continuously improve output efficiency while also contributing to the economy's and society's long-term, sustainable growth. Due to the integrated development of digital technology and the sports industry, the application of digital technology can promote the structural upgrading, process optimization, supply and demand matching, and business integration of the sports industry, as well as improve resource utilization efficiency while reducing the carbon emissions of the sports industry unit GDP, and then influence and control the sports industry. As a result of the process of linear scale expansion, total carbon emissions have increased. By integrating the most advanced digital technologies, such as the Internet of Things and artificial intelligence, into the venue's construction and operation, and by promoting energy efficiency through intelligent control of lighting and temperature, as well as energy consumption, the venue can achieve low-carbon operations while preventing energy waste. The sporting goods manufacturing industry has also been impacted by digital technologies, such as the Internet of Things and artificial intelligence, which has prompted the industry to continuously integrate product manufacturing with product R&D and design, as well as raw material procurement, warehousing, and transportation at the front end of the industry chain and product branding and channel marketing services at the back end. This transformation into a manufacturing company focused on an ongoing service. On the basis of these factors, the continued integration of digital technology into the sports industry will continue to promote the green development of the sports industry due to the efficiency improvement and low-carbon advantages that digital technology offers.

The article "Development Analysis of the Sports Industry Based on the Data Mining Model" was published in 2022. Journal: Comput Intell Neurosci.

### 2.3. Strategy

Fundamental to sustainable development in the sports business is promoting the green growth of that industry. This is the overarching objective of the green development in the sports industry. In the sports industry, green refers to the regulatory framework that governs the specific technique of development used, while development refers to the end aim that the sports sector must reach. It is necessary to adopt it broadly throughout the sports industry system in order to support the green growth of the sports industry. Green growth management is the management of green growth. In conjunction with the current state of the green development of the sports industry, the green transformation of the sports goods manufacturing industry and the expansion of the scale of the sports service industry are the two most important directions for the green development of the sports industry going forward.

The sporting goods manufacturing business has a close industrial relationship with the rest of the world. Upstream and downstream industrial chains in the country are not only linked to agricultural production, such as cotton, in the primary industry, but they are also linked to industrial production, such as textiles and rubber, steel, and construction, in the secondary industry, and even linked to the tertiary industry, such as warehousing, logistics, sales, packaging, and other modern services, that are also provided in the country. Additionally, the manufacturing process and the production method used by the sporting goods manufacturing industry must consume a significant amount of natural resources, energy, and industrial water, while also producing a significant amount of solid waste and greenhouse gases as a result of their operations. Furthermore, as a result of the misalignment between supply and demand, a large number of primary sporting goods are frequently left idle or disposed of at low prices, resulting in resource waste and a failure to improve the resource productivity and carbon productivity of the sporting goods manufacturing sector. It is necessary to change the development mode of the sports goods manufacturing industry in order to promote the realization of green and clean production in order to green the sports goods manufacturing industry. For the sports industry to achieve green production, the sports manufacturing production department must continuously improve the design concept, technical process, and energy consumption; it must also continuously reduce energy consumption in the manufacturing process; it must reduce the intensity with which natural resources and intermediate inputs are used; and it must reduce carbon dioxide and pollutant emissions.

The article "Development Analysis of the Sports Industry Based on the Data Mining Model" was published in 2022. Journal: Comput Intell Neurosci.

The development and growth of the sports service industry can not only increase the linear growth of the added value of the sports service industry but it can also optimize the internal structure of the sports service industry and promote the development of the sports service industry that is environmentally friend and low in carbon emissions. It is imperative that the scale and level of industrialization be raised as soon as possible. A high economic output, little resource consumption, and low-carbon emissions are all required for the industrialization of the life sports service industry. In order to provide industrialization, scale, and branding, the main body of life sports services is being accelerated to become more market-oriented, relying on professional management processes, and standards to provide serialized and personalized sports services, through the effective supply of sports services to expand and promote sports consumption, forming economies of scale and scope.

It is essential that the provision of fitness and leisure services, the integration of sports and education under the umbrella of active health needs, as well as the physical education and training made possible by the reform of the sports examination system, and continued to contribute to the resolution of major social needs and important social concerns. The efficient provision of sports services will hasten the industrialization and expansion of the sporting goods and services industry. To achieve economies of scale and scope in the sports service industry, it is vital to accelerate the adoption of digital technologies in this sector as soon as possible. Strengthening the digitalization of the sports service industry will help to ensure that sports services are oriented on the demands of sports consumers, that new models and new formats are progressively formed, and that the value creation is promoted. As a result, it can help to boost industry integration and industrial chain collaboration while also improving industrial efficiency on a continual basis in the sports service industry. In addition, the configuration of parts should be optimized. Businesses' marginal costs can be greatly reduced as a result of the increased use of digital technology in their operations. Sports service providers can raise the number of consumers they serve, expand their business scope, enhance related earnings, establish economies of scale and scope, and progressively solve the current sports challenges by utilizing deep data processing. The dilemma of service entities having a narrow output scale and a limited ability to drain their resources. Finally, in order to increase the overall quality of the provision of sports services, it is required to tighten market monitoring. With rapid growth came the exposure of negative business practices, such as infringement of consumer rights and interests and misappropriation of consumer assets. This resulted in a significant decrease in consumers' confidence and enthusiasm for the sports, fitness, and leisure industries, as well as the physical education and training industry. However, there are still significant shortcomings in the overall supervision regulations as well as the performance of supervision responsibilities in the current sports market, and the supervision subjects and supervision behaviors of the subdivided market are still out of the question in the current sports market. The need for increased market oversight of sports services, as well as improved quality of sports service supply, is therefore critical at this point of time.

The article "Development Analysis of the Sports Industry Based on the Data Mining Model" was published in 2022. Journal: Comput Intell Neurosci.

## 3. The Proposed Model

In this chapter, we propose a data mining method to analyze the development of the sports industry. The global steady-state feature fusion strategy is used to realize the construction of a distributed time series model of sports industry data in order to realize the construction of an accurate time series-based mining model of sports industry data. Together with semantic ontology fusion, the underlying data module creates a spatial distribution structural model of sports data. Using the spatial distribution structure feature matching method, the compatibility feature distribution concept set of sports industry data is generated.

(1) $$\begin{array}{c} \text{Sim}\left(Q_{n},R_{n}\right)=\alpha \text{Sim}\left(Q_{n+1},R_{n+1}\right)+\text{Sim}\left(A_{Q_{n}},A_{R_{n}}\right), \end{array}$$

where *α* is the fusion parameter of the leaf node of the sports industry data spatial distribution structure, and the state parameter of the central node is introduced to obtain the ith sports industry. Data spatial distribution attribute, *A*_*Q*_*n*__, *A*_*R*_*n*__ is the fuzzy state feature quantity of the central node of the sports industry data spatial distribution structure, *Q*_*n*+1_, *R*_*n*+1_ are the joint feature solutions in the current sports industry data spatial distribution structure, according to the above distribution structure design, according to the similarity between attribute nodes and attribute value nodes, the stable feature analysis method of sports industry data mining is obtained, and the nonlocal integral-differential singular vector is obtained. Under the finite overall distribution, the convergence state equation of sports industry data mining is obtained as

(2) $$\begin{array}{c} C=u\sum_{i=1}\text{Sim}\left(Q_{n},R_{n}\right), \end{array}$$

where *u* represents the degree of association of nodes in the spatial distribution model of sports industry data. Using nonlocal singular disturbance constraints, the eigenvalues of periodic solution are output, and the constraints of the integrodifferential equations for the distribution of sports industry data is

(3) $$\begin{array}{c} Q=e\times C, \end{array}$$

where *e* represents the nonlocal singular perturbation constraint value. In the terminal sliding mode surface, the similar feature quantities of the obtained subconcept map are expanded as follows:

(4) $$\begin{array}{c} F=c\left(A_{Q_{n}},A_{R_{n}}\right)+u. \end{array}$$

When it comes to realizing the quantitative spatial transformation of sports industry data, the statistical and quantitative fusion analysis method is used, and the correlation distribution of sports industry data is mined using the fuzzy analytical control method, which results in the following deep learning model for the correlation evaluation of sports industry data.

(5) $$\begin{array}{c} R=\delta \sum T_{rj}+\alpha . \end{array}$$

Using the similarity feature analysis method, the correlation dimension distribution structure feature of sports industry data is obtained. Based on the model design method of a recursive algorithm, the optimal feature amount of sports industry data mining is obtained as *T*_*rj*_. Taking the recursive concept map as the semantic feature solution, we get the adaptive parameter fusion model of sports industry data mining *σ*_*i*_(*k*), when *i* = 1, adopt recursive concept map analysis to obtain the matching calculation result *u*_*i*_ of sports industry data, which satisfies the convergence condition *α*_*ri*_(*k*).

The article "Development Analysis of the Sports Industry Based on the Data Mining Model" was published in 2022. Journal: Comput Intell Neurosci.

The fitness function evaluation value of sports industry data mining can be obtained from the recursive formula:

(6) $$\begin{array}{c} W=\sum_{k=1}\text{ln}\left(\frac{1}{u_{i}}\times \frac{{\left|\alpha_{n}\left(k\right)\right|}^{2}}{\sigma_{i}\left(k\right)}\right)+R. \end{array}$$

And we have

(7) $$\begin{array}{c} u_{j}^{\prime \prime }=p_{rj}\left(k\right)-\sum_{k=1}^{\eta }\ln\left(\frac{1}{u_{i}}\times \frac{{\left|\alpha_{n}\left(k\right)\right|}^{2}}{\sigma_{i}\left(k\right)}-1\right), \end{array}$$

where *p*_*rj*_(*k*) is the optimal value of the joint probability density of sports industry data distribution. According to the similarity distribution of the two structure pairs [10], the information fusion clustering processing of sports industry data mining is carried out, and the fuzzy evaluation function of the information fusion is obtained as

(8) $$\begin{array}{c} y_{i}^{\prime }=u_{i}^{\prime \prime }T_{rj}+n_{i}, \end{array}$$

where *n*_*i*_ is the joint matching function of the concept map CQ and the concept map CR.

Using the output gain steady-state analysis method, a linear analytical parameter analysis model for sports industry data mining is constructed, and the concept map's central parameters (CR) are obtained by applying the square programming and linear fusion methods to the concept map's central parameters (CR) [10]. Then we have

(9) $$\begin{array}{c} {\text{Sim}}_{y}\left(y_{1},y_{2}\right)=\text{Typc}\left(y_{1},y_{2}\right). \end{array}$$

Using the linear fusion method of sports industry data mining and the distributed joint control function of attribute value nodes for sports industry data evaluation, the distributed joint control function of attribute value nodes for sports industry data evaluation is created. After analyzing all typical solutions, the output joint reliability distribution function of sports industry data mining is determined. In the sports industry, data mining has produced some interesting statistics. This is the feature quantity, and the binary linear programming model for precise mining of sports industry data satisfies the following conditions in all corresponding E-A models.

(10) $$\begin{array}{c} U=\sum \sum \ln\left(\frac{1}{\gamma }\frac{{\text{Sim}}_{y}\left(y_{1},y_{2}\right)}{\sigma_{i}{\left(k\right)}^{2}}-1\right). \end{array}$$

The convergence condition of the mining output satisfies

(11) $$\begin{array}{c} J=\int \left(K\times f\left(x_{1},x_{2},i\right)\right)x\text{d}u+\alpha_{ri}. \end{array}$$

Based on the above analysis, combined with the sparse feature matching scheduling model, the time fusion sequence of sports industry data mining is constructed, and the accurate mining of sports industry data is realized through time series reconstruction.

The article "Development Analysis of the Sports Industry Based on the Data Mining Model" was published in 2022. Journal: Comput Intell Neurosci.

## 4. Results

This paper collects the data of three sports companies and divides 75% of the sports industry data of these companies into the training set and the remaining 25% into the test set in order to evaluate the application performance of the method presented in this paper in achieving accurate data mining in the sports industry. Matching coefficient (MC) and reliability (*E*) are selected as evaluation indicators. The method of calculating *E* is as follows:

(12) $$\begin{array}{c} E_{i}=\frac{\left|{\text{Sim}}_{i}-{\text{Sub}}_{i}\right|}{{\text{Sim}}_{i}}\times 100\%. \end{array}$$

For the fairness of the comparison, the parameters used in the algorithm in this paper are consistent with those in Reference 6. Our comparison algorithms are FK-means, PSO, and DDM. First, we compared the convergence curves between different models, as shown in Figure 1.

The analysis of Figure 1 reveals that the method presented in this paper has superior convergence for data mining in the sports industry, while the FK-means and PSO methods have slower convergence rates and the DDM has faster convergence rates than PSO and FK-means. Figures 2 and 3 illustrate the results of a comparison of the matching degree and index of reliability of various data mining techniques for the sports industry.

In terms of algorithm complexity, since this paper does not introduce additional parameters, it does not increase the algorithm complexity.

It can be seen from Figures 2 and 3 that the algorithm proposed in this paper is better than KF-means, PSO, and DDM in terms of matching degree and reliability. In addition, among the four algorithms, the KF-means algorithm has the worst performance, and DDM is inferior to our algorithm.

Further, this paper tests the robustness of the proposed method. We add noise to the sports industry-related data set to the test whether the MC and E of the algorithm are still robust. After adding a certain noise that obeys the normal distribution, the MC of the method in this paper is 0.798, and the E is 0.81. Although it is lower than the test result without noise, it still shows that the method in this paper is robust.

## 5. Conclusion

The big data business in sports has reached a point of maturity and utility, presenting new opportunities and challenges for the development of Chinese sports. While seizing opportunities, it is essential to comply with sports and big data development laws. China's sports big data is in its exploratory phase; therefore, it is essential to examine its integrated development model in order to assist businesses in identifying advantageous implementation and application areas. Future growth of the sports big data industry will present additional obstacles. Only by integrating with China's national conditions and resolving them with cross-border thought and inventiveness will we be able to continuously advance sports big data.

The article "Development Analysis of the Sports Industry Based on the Data Mining Model" was published in 2022. Journal: Comput Intell Neurosci.

China's sports sector is a diversified industry that incorporates the country's secondary and tertiary industries. The issues of unbalanced industrial structure development, mismatch between supply and demand, and rapid expansion in the sports goods manufacturing industry are becoming increasingly prominent. The objective of this study is to first examine the dynamic mechanism and promotion strategy for the green development of the China's sports industry by conducting a literature review. In addition, a time series-based sports industry data analysis model is provided in order to improve the precision of data mining and quantitative analysis in the sports industry. In order to achieve precise data mining in the sports industry, the global steady-state feature fusion method, the statistical and quantitative fusion analysis method, and the fuzzy analytical control method are utilized. Simulation results indicate that this method is more precise and has a higher level of feature matching for sports industry data mining, thereby reducing the disturbance error associated with sports industry data mining.

## Figures and Tables

**Figure 1:** Comparison of convergence speeds of different methods.

**Figure 2:** Comparison of MC.

**Figure 3:** Comparison of E.

## Data Availability

The data used to support the findings of this study are available from the corresponding author upon request.

## References

[1] Wu Z., Zhou C. (2021). Construction of an intelligent processing platform for equestrian event information based on data fusion and data mining. *Journal of Sensors*.

[2] Hao L. I. U. (2016). A score management system design for sports using data mining: analysis of a new study[J]. *International Journal of Simulation. Systems, Science and Technology*.

[3] Rajšp A., Fister I. (2020). A systematic literature review of intelligent data analysis methods for smart sport training. *Applied Sciences*.

[4] Cui Z., Yan C. (2020). Deep integration of health information service system and data mining analysis technology. *Applied Mathematics and Nonlinear Sciences*.

[5] Liou J. J. H., Chang M.-H., Lo H.-W., Hsu M.-H. (2021). Application of an MCDM model with data mining techniques for green supplier evaluation and selection. *Applied Soft Computing*.

[6] Li H. (2020). Analysis on the construction of sports match prediction model using neural network. *Soft Computing*.

The article "Development Analysis of the Sports Industry Based on the Data Mining Model" was published in 2022. Journal: Comput Intell Neurosci.

[7] Li H. Trend analysis of university sports venues opening to outside world based on big data[C].

[8] Thongtae P., Srisuk S. An analysis of data mining applications in crime domain[C].

[9] Das D., Shorif Uddin M. (2013). Data mining and neural network techniques in stock market prediction: a methodological review. *International journal of artificial intelligence & applications*.

[10] Chen F., Deng P., Wan J., Zhang D., Vasilakos A. V., Rong X. (2015). Data mining for the Internet of Things: literature review and challenges. *International Journal of Distributed Sensor Networks*.

[11] Schumaker R. P., Solieman O. K., Chen H. (2010). *Sports Data mining[M]*.

[12] Parmezan Bonidia R., Duilio Brancher J., Marques Busto R. (2018). Data mining in sports: a systematic review. *IEEE Latin America Transactions*.

[13] Zhang L. (2020). Design of a sports culture data fusion system based on a data mining algorithm. *Personal and Ubiquitous Computing*.

[14] Haghighat M., Rastegari H., Nourafza N. (2013). A review of data mining techniques for result prediction in sports[J]. *Advances in Computer Science: An International Journal*.

[15] Rojas-Valverde D., Gómez-Carmona C. D., Gutiérrez-Vargas R. (2019). From big data mining to technical sport reports: the case of inertial measurement unit. *BMJ open sport & exercise medicine*.

[16] Schumaker R. P., Solieman O. K., Chen H. (2010). Sports knowledge management and data mining. *Annual Review of Information Science & Technology*.

[17] Song W., Xu M., Dolma Y. (2019). Design and implementation of beach sports big data analysis system based on computer technology. *Journal of Coastal Research*.

[18] Yang K. (2020). The construction of sports culture industry growth forecast model based on big data. *Personal and Ubiquitous Computing*.

[19] Schoeman J. H., Matthee M. C., Van Der Merwe P. (2006). The viability of business data mining in the sports environment: cricket match analysis as application[J]. *South African Journal for Research in Sport, Physical Education and Recreation*.

[20] Liu H. (2019). Opportunities, challenges and Countermeasures for the development of China’s sports industry in the era of big data. *Journal of Physics: Conference Series*.

[21] Xun G., Suxia L. (2018). Construction of evaluation system of sports talent training scheme based on data mining. *International Journal of Reasoning-based Intelligent Systems*.

